The article "Differential temporal expression of S100β in developing rat brain" was retracted in 2023. Reasons: unreliable data; unreliable results or conclusions; concerns about the images.

# Differential temporal expression of S100β in developing rat brain

**DOI:** 10.3389/fncel.2015.00087

**Published:** 2015-03-18

**Authors:** Nisha Patro, Aijaz Naik, Ishan K. Patro

**Affiliations:** ^1^School of Studies in Neuroscience, Jiwaji University Gwalior, India; ^2^School of Studies in Zoology, Jiwaji University Gwalior, India

**Keywords:** S100β, nestin, GFAP, astrocyte, neural development

## Abstract

Radial glial cells (RGs) originally considered to provide scaffold to the radially migrating neurons constitute a heterogeneous population of the regionally variable precursor cells that generate both neurons as well as glia depending upon the location and the timing of development. Hence specific immunohistochemical markers are required to specify their spatiotemporal location and fate in the neurogenic and gliogenic zones. We hypothesize S100β as a potential and unified marker for both primary and secondary progenitors. To achieve this, cryocut sections from rat brains of varied embryonic and postnatal ages were immunolabeled with a combination of antibodies, i.e., S100β + Nestin, Nestin + GFAP and S100β + GFAP. A large population of the primary and secondary progenitors, lining the VZ and SVZ, simultaneously co-expressed S100β and nestin establishing their progenitor nature. A downregulation of both S100β and nestin noticed by the end of the 1st postnatal week marks their differentiation towards neuronal or glial lineage. In view of the absence of co-expression of GFAP (glial fibrillary acidic protein) either with S100β or nestin, the suitability of accepting GFAP as an early marker of RG’s was eliminated. Thus the dynamic expression of S100β in both the neural stem cells (NSCs) and RGs during embryonic and early neonatal life is associated with its proliferative potential and migration of undifferentiated neuroblasts and astrocytes. Once they lose their potential for proliferation, the S100β expression is repressed with its reemergence in mature astrocytes. This study provides the first clear evidence of S100β expression throughout the period of neurogenesis and early gliogenesis, suggesting its suitability as a radial progenitor cell marker.

## Introduction

Radial glia are the primary progenitor cells during early embryonic neurogenesis with a capacity to generate all types of neurons and glia (Noctor et al., 2001, 2002; Tamamaki et al., 2001; Rowitch and Kriegstein, 2010). Similar to the neuroepithelial cells from which they are derived the radial glia progenitors (RGP), also line the ventricular zone (VZ), maintain an apico-basal polarity, extend processes radially from the VZ to the pial surface, exhibit interkinetic nuclear migration and divide asymmetrically to self-renew and either to generate a post-mitotic neuron/glia or intermediate progenitor cell (IPC; Tamamaki et al., 2001; Malatesta et al., 2003; Anthony et al., 2004; Haubensak et al., 2004; Miyata et al., 2004; Noctor et al., 2004, 2008; Götz and Huttner, 2005). The radial glia are now considered to be a dynamic, multifaceted cell type that persists and changes its role in response to signals from the surroundings throughout the organism’s life (Sild and Ruthazer, 2011). In addition to the VZ, the embryonic sub ventricular zone (SVZ) having cells derived from RG is also considered as a major site for neurogenesis (Noctor et al., 2001, 2004, 2008; Tarabykin et al., 2001; Smart et al., 2002; Nieto et al., 2004; Zimmer et al., 2004; Pontious et al., 2008; Kriegstein and Alvarez-Buylla, 2009). Earlier the SVZ was considered to be a site of gliogenesis only (Altman and Bayer, 1990; Takahashi et al., 1995). Subsequent imaging studies on the divisions of precursor cells within the SVZ have demonstrated their neurogenic potential (Miyata et al., 2004; Noctor et al., 2004).

The article "Differential temporal expression of S100β in developing rat brain" was retracted in 2023. Reasons: unreliable data; unreliable results or conclusions; concerns about the images.

Radial glia were so named as they present many glial properties including expression of glial markers like glial fibrillary acidic protein (GFAP) and astrocyte specific glutamate transporter (GLAST; Levitt and Rakic, 1980; Campbell and Götz, 2002). Hence RGs are considered to be the astrocyte precursors performing astrocyte like functions and subsequently transforming into astrocytes (Cajal, 1909; Schmechel and Rakic, 1979; Voigt, 1989; Tramontin et al., 2003). Embryonic neural stem cell (NSC) properties of these cells were subsequently demonstrated based on Cre-recombinase gene expression in a Cre/loxP fate mapping using the radial glia specific brain lipid binding protein (BLBP) promoter to drive the expression of Cre and the labeling of a large number of neurons in all brain regions (Anthony et al., 2004).

Nestin, a class VI intermediate filament protein is expressed in the majority of mitotically active CNS and PNS progenitors that give rise to both neurons and glia (Lendahl and McKay, 1990; Mujtaba et al., 1998; Michalczyk and Ziman, 2005) and is downregulated in cells upon differentiation (Zimmerman et al., 1994; Lothian and Lendahl, 1997; Sahlgren et al., 2001). Thus nestin is used as a widely accepted marker of NSCs having self-renewal ability (Lendahl and McKay, 1990). RG cells now considered to be potential precursor cells also express nestin (Parnavelas and Nadarajah, 2001). However, there are reports in the literature indicating the re-expression of nestin during various regenerative and degenerative conditions in fully differentiated cells (Geloso et al., 2004; Corvino et al., 2005).

The article "Differential temporal expression of S100β in developing rat brain" was retracted in 2023. Reasons: unreliable data; unreliable results or conclusions; concerns about the images.

In rodents, phenotypes of the primary RG cells can be recognized by immunoreactivity to radial glial cell marker 1 (RC1; Edwards et al., 1990), radial glial cell marker 2 (RC2; Misson et al., 1988a), Vimentin (Schnitzer et al., 1981; Pérez-Álvarez et al., 2008), GLAST (Shibata et al., 1997), Rat 401 (Colombo and Napp, 1996), Ran-2 (Bartlett et al., 1981), BLBP (Feng et al., 1994), etc. However, the neuroepithelial cells do not express many of these markers. RG cells are GFAP−ve in rodents till the completion of corticogenesis and the vimentin is substituted to GFAP during emergence of secondary phenotype (Bovolenta et al., 1984; Misson et al., 1988a,b; Cameron and Rakic, 1991). The GFAP immunoreactivity in RG’s in rodents can be observed only after birth (Rakic, 2003). In both human and monkey cerebral cortex the RG cells have been reported to transform into fibrillary astrocytes and/or protoplasmic astrocytes (Rakic, 1978, 1995; Schmechel and Rakic, 1979; Levitt and Rakic, 1980; Rickmann et al., 1987; Voigt, 1989). The time of disappearance of RG cells in the neocortex, hippocampus and cerebellum correlates well with the appearance of astrocytes in these brain areas (Rakic, 1971, 1972; Schmechel and Rakic, 1979; Eckenhoff and Rakic, 1984). This coincides with the downregulation of RC1, RC2 and Rat-401 antigens, which are never re-expressed in adult brain (Misson et al., 1988a,b; Evrard et al., 1990) and a concomitant and gradual appearance of GFAP expression (Culican et al., 1990; Misson et al., 1991).

In addition S100β is also commonly used as a marker of Bergmann glia in the cerebellum of adult rodents (Landry et al., 1989; Patro et al., 2009). However, Vives et al. (2003) reported that the S100β gene was activated during histogenesis of the cerebellum between E13.5 to P3. They also noted the presence of a large population of S100β expressing cells and assumed them to be immature Bergmann glial cells. Subsequently, Hachem et al. (2007) marked the activation of S100β gene in radial glial precursors as a feature of Bergmann cell gliogenesis. In view of this and the role of S100β in the regulation of proliferation, differentiation and phenotyping of neurons (Donato, 2001, 2003; Santamaria-Kisiel et al., 2006; Donato et al., 2009, 2013) it was worthwhile to investigate if S100β could be a marker for radial glial progenitors or the neural progenitors as a whole in the developing brain which are actively proliferating.

The present study hypothesizes S100β as a specific and unified marker for both the neuroepithelial (primary progenitor cells) and RG cells in the ventricular and subventricular zone throughout the period of embryonic and early neonatal life. The results also indicate possible role of S100β in maintaining the proliferative potential of these cells. The protein is repressed during second week of postnatal life and reappears and is expressed in the mature astrocytes.

The article "Differential temporal expression of S100β in developing rat brain" was retracted in 2023. Reasons: unreliable data; unreliable results or conclusions; concerns about the images.

## Material and Methods

### Tissue Preparation for Immunohistochemical Studies

Naive Sprague Dawley female rats (200–225 g, 3 month old) were housed in our animal house facility under standard laboratory conditions, viz., a standard light/dark cycle of 12 h (7 am–7 pm), room temperature of 23 ± 2°C and *ad libitum* access to pellet food and water. Timed pregnancies were set and confirmed in the dams by a 4 h pairing with breeder males followed by vaginal smear examination. For harvesting the embryos of varied embryonic age, viz., E11, 14, 16 and 18, timed pregnant females were sacrificed on the respective days and embryos were removed. For E11, the whole embryo was processed while for E14, 16 or 18 days (*n* = 3) the brains were micro-dissected from the embryos with sterilized and atraumatic instruments and fixed in 2% phosphate buffered paraformaldehyde (PFA; pH 7.4), cryoprotected in phosphate buffered sucrose gradients (10%, 20%, 30%) and sagittal sections were cut.

For postnatal brain tissue harvesting timed pregnant dams were observed carefully every 2 h on the expected days of delivery to mark the day of birth as postnatal day 0 (P0). Pups were housed with their mothers in individual cages until weaning at P21. On various postnatal study time-points (P2, 5, 12, 15, 21 and 30; *n* = 3), the pups were deeply anesthetized and perfusion-fixed, transcardially with ice-cold saline followed by 2% PFA in 0.1 M PBS (pH 7.4). The brains were dissected out, post-fixed overnight with 2% PFA and subsequently cryoprotected with sucrose gradients (10%, 20%, 30%) prepared in 0.1 M PBS, pH 7.4.

Sections of 15 μm thickness were cut with the help of Leica Cryotome (CM1900; Germany) and collected on chromalum gelatin coated slides. For embryonic brains the sections were cut sagittally while for postnatal brains the coronal sections were cut through the occipito-temporal region. The sections were then stored at −20°C to be used for immunohistochemical studies. All the experiments were pre-approved by the Institutional Animal Ethics Committee and performed as per the strict instructions and guidelines of CPCSEA (Committee for the purpose of control and supervision on experiments on animals). All efforts were made to minimize the sufferings caused to the animals and to reduce the number of animals used.

### Immunohistochemistry and Fluorescence Microscopy

#### Nestin + S100β Co-Labeling

Nestin and S100β dual labeling was done to emphasize the stem cell nature of the RG and to further examine if they do express S100β as well. This was achieved by employing the sequential staining protocol for dual immunolabeling. Brain sections containing either VZ or SVZ and subgranular zone (SGZ) were carefully selected randomly from amongst the pooled sections (of each age group) from all the embryos/pups of various age groups, viz., E11, E14, E16, E18 P0, P2, P5, P12, P21 and P30 and air-dried at room temperature. After drying, the sections were washed thrice (5 min each) with phosphate buffered saline (0.1 M; pH 7.4) to remove cryomount. The sections were then incubated with 0.5% triton X-100 (Sigma) in PBS for 20 min to ensure membrane permeabilization. This was followed by washings of 5 min each with PBST (PBS containing 0.1% Tween-20). Incubating sections in 10% normal goat serum in PBS blocked non-specific proteins for 90 min at room temperature. The sections were first incubated with Mouse anti-Nestin (Chemicon; MAB 353) at a titer of 1:100, diluted with 5% BSA in PBST at 4°C overnight. Next day the sections were washed with 3 changes of PBST (5 min each) and further incubated with anti-mouse FITC conjugated secondary antibody (Sigma) for nestin detection. For completely eluting the primary and secondary antibodies from the first staining, the sections were rigorously washed in PBS (5 × 10 min) and incubated with 10% normal goat serum in PBS for 2 h at room temperature. Subsequently the sections were incubated with second primary antibody, Mouse monoclonal anti- S100β (Sigma, 1:500; S 2532), overnight at 4°C and then detected with anti-mouse TRITC conjugated (Sigma) secondary antibody. All antibody dilutions were made in 5% Bovine Serum Albumin (BSA) in PBST. The sections were then washed with PBS (5 × 10 min) and mounted in an aqueous mounting medium from Vector Laboratories, Vectashield Hardset with DAPI.

The article "Differential temporal expression of S100β in developing rat brain" was retracted in 2023. Reasons: unreliable data; unreliable results or conclusions; concerns about the images.

#### Nestin + GFAP and GFAP + S100β Co-Labeling

Simultaneous staining protocol was opted by using unlabelled primary antibodies from different host species. The sections after membrane permeabilization and protein blocking were incubated with cocktail of Mouse anti-Nestin (Chemicon) and Rabbit anti-GFAP (Dako, 1:1000; Z 0334) or Rabbit anti-GFAP and Mouse S100β antibodies for overnight at 4°C. Antigen detection was done, by incubating in an appropriate fluorochrome conjugated secondary antibody mixture, viz., anti-mouse FITC and anti-rabbit TRITC for Nestin + GFAP and anti-Rabbit FITC and anti-Mouse TRITC for GFAP + S100β. Anti-GFAP antibody was used at a concentration of 1:1000 diluted in 5% BSA in PBST.

In order to avoid any unexpected inter-species cross-reactivity, all the secondary antibodies raised in the same host, were used. All antibody dilutions were made in 5% BSA in PBST. Finally the sections after thorough washing in PBS were mounted in aqueous mounting medium from Vector Laboratories, Vectashield Hardset with DAPI. Some sections were used as negative controls by omitting the primary antibody. No specific staining was observed in these sections. To maintain comparability in developmental profiling of the various markers used, all the tissues were processed and stained in parallel. Prior to co-localization by sequential or simultaneous methods, the antibodies were also tried individually in the same brain sections and similar results were obtained by either of the procedures.

The images were acquired in a manner blinded to the investigator(s) with the help of Leica DM 6000 Fluorescence microscope using appropriate filters and LAS AF (Leica Application suite Advanced Fluorescence) imaging software. Identical conditions were applied for microscopy and image processing.

## Results

### S100β as a Radial Progenitor Cell Marker

To visualize the radial glial progenitor cells in the developing rat brain during the embryonic and postnatal life, we used a monoclonal antibody against nestin, a well-established marker known to label both the NSCs/neuroepithelial cells and radial glial progenitor cells (Lendahl and McKay, 1990; Parnavelas and Nadarajah, 2001). The antibody labeled both the primary progenitor/neuroepithelial stem cells and radial glia/secondary progenitor cells lining the VZ at early embryonic age (E11 and E14; Figures 1A,B,E,F respectively) and subventricular zone (SVZ) during late embryonic and early neonatal life. By E16, most of the nestin labeled radial glial fibers were confined to the SVZ (Figures 1I,J).

**Figure 1:** **S100β labels both primary and secondary progenitors at VZ and SVZ during early embryonic life**. Sagittal sections through the developing forebrain were co-immunostained with antibodies against Nestin (green) and S100β (red). All the progenitors lining VZ and SVZ were strongly positive for Nestin **(B,F,J)** and S100β **(C,G,K)**. A strong co-localization of both the markers was detected at VZ **(D,H)** and SVZ **(L)** zones. DAPI (blue) clearly indicated the brain areas focused **(A,E,I)**.

While S100β has been well reported to have a role in proliferation and differentiation and a marker of mature astrocytes, Haubensak et al. (2004) reported it’s expression in primary radial glial scaffolds involved in Purkinje progenitor exit from the VZ. They correlated S100β expression in RGs of the cerebellar VZ, with the onset of gliogenesis.

This observation incited us to use S100β as a radial glial marker. Interestingly when we did dual immunofluorescence labeling with nestin and S100β, the merged images clearly depicted that all the nestin labeled cells in the VZ of E11 and E14 brains were S100β+ve as well. This was true for both the primary progenitors/neuroepithelial cells as well as the secondary progenitors/radial glial cells. Similar to nestin immunoreactivity, radial glial cells with their glial scaffold extending from VZ to pial surface were well labeled with S100β (Figures 1C,G). Both the nestin and S100β expression coincided perfectly in the overlay images (Figures 1D,H).

The article "Differential temporal expression of S100β in developing rat brain" was retracted in 2023. Reasons: unreliable data; unreliable results or conclusions; concerns about the images.

Around birth (P0), the nestin labeled radial fibers were radically reduced in number and the nestin+ progenitors having radial morphology were seen mainly lining the SVZ and SGZ (sub granular zone) only (Figures 2A,B,E,F). By the end of the second postnatal week the nestin+ progenitor cells disappeared gradually indicating their differentiation into specific cell types in the mature hippocampus. In addition, the S100β also labeled the radial glial progenitors of the SVZ in E16 embryonic brains (Figure 1K) and well matched the expression of nestin in merged images (Figures 1, 2). Similarly in the early neonatal brains also, all the nestin labeled progenitors were S100β+ as well (Figures 2C,D,G,H), clearly indicating that S100β similar to nestin also act as a marker for stem cells or progenitors having multiple phenotypes. The nestin+ stem astrocytes at P2 forming glial tubes co-expressed S100β (Figures 2I–L), indicating their stem cell nature. However, at weaning age, i.e., P21 the S100β was expressed in mature astrocytes with no nestin positivity (Figures 2M–P).

**Figure 2:** **S100β labels the progenitors both at SVZ and SGZ around birth and is re-expressed in mature astrocytes**. Dual immunofluorescence labeling with Nestin (green; **B,F,J,N**) and S100β (red; **C,G,K,O**). The expression of both the markers coincided completely in the radial fibers and progenitors at SVZ **(D)** and SGZ **(H)** around birth. At P2 the stem astrocytes forming glial tubes (arrows) were labeled for both Nestin and S100β **(L)**. Mature astrocytes loose Nestin and express S100β only **(O)**. In merged image at P30 **(P)** no S100β labeled astrocytes co-expressed Nestin. DAPI (blue) clearly indicated the brain areas focused **(A,E,I,M)**.

### Nestin + GFAP

Adult NSCs express GFAP and nestin both along with other astrocytic features and are thus named as stem astrocytes (Seri et al., 2004; Steiner et al., 2006). Nestin + GFAP colabeling in the developing brain would help us to know the status of the neural progenitors and differentiate them from the adult stem cells.

The article "Differential temporal expression of S100β in developing rat brain" was retracted in 2023. Reasons: unreliable data; unreliable results or conclusions; concerns about the images.

Surprisingly, throughout the embryonic life (E11–E18), none of the nestin+ progenitors and radial glia co-expressed GFAP (Figures 3A–D), although GFAP expression was first localized at E16 in the hippocampal niche close to SVZ (Figure 5F). Following this there was a gradual increase in the GFAP+ astrocyte population in brain areas in the vicinity of SVZ. But one of these GFAP expressing astrocytes co-expressed nestin. Even at P0 the radial glia of the SVZ (Figures 3E,F) and the bipolar progenitors lining the sub granular zone (SGZ) were nestin+ only (Figures 3I,J) and did not express GFAP at all (Figures 3G,H,K,L). Only at P2, adult SVZ astrocytes forming the glial tubes in the neocortical SVZ (Figure 4A), were expressing both the nestin and GFAP (Figures 4B,C), thus, displaying the features of the radial/stem astrocytes. The expression of GFAP coincided with that of nestin in most of these stem astrocytes in merged images (Figure 4D). Such radial astrocytes forming glial tubes depicted the chain migration of stem astrocytes, tangentially along the corpus callosum and neocortex. Subsequently by P5 some of the progenitors lining the SVZ and SGZ co-expressed both nestin and GFAP, while others were either nestin or GFAP+ve only (Figures 4E–L). By 2nd and 3rd week the number of nestin+ progenitors (Figure 4N) decreased gradually with a simultaneous increase in the GFAP+ and morphologically mature astrocytes (Figure 4O). By P21 the astrocytes expressing both nestin and GFAP were very occasional (Figures 4M–P).

**Figure 3:** **No GFAP expression in the Radial progenitors at SVZ and SGZ during embryonic life and around birth**. Immunofluorescence staining for DAPI (blue; **A,E,I**), Nestin (green; **B,F,J**) and GFAP (red; **C,G,K**). Merged images are shown in **(D), (H)** and **(L)**. Radial glia and progenitors uniformly express nestin throughout the embryonic and early neonatal life. No GFAP co-immunostaining with nestin was observed.

**Figure 4:** **Stem astrocytes forming the glial tubes in neocortical SVZ and at SGZ co-express Nestin and GFAP**. Immunofluorescence staining for DAPI (blue; **A,E,I,M**), Nestin (green; **B,F,J,N**) and GFAP (red; **C,G,K,O**). Merged images are shown in **(D), (H), (L)** and **(P)**. Stem astrocytes forming the glial tubes in the neocortical SVZ (arrows; **D**) and those lining the SGZ and SVZ co-express Nestin and GFAP **(H,L)**. Mature astrocytes at P21 express only GFAP and no Nestin staining was detected **(P)**.

**Figure 5:** **S100β labels the progenitors during embryonic and early neonatal life and differentiated astrocytes at adulthood**. Double immunostaining with GFAP (green; **B,F,J,N**) and S100β (red; **C,G,K,O**) reveals appearance of GFAP at hippocampal niche at E16 (arrows; **F**) while uniform S100β staining in the VZ at E11 **(C)** and SVZ at E16 **(G)**. At P0 a further increase in GFAP immunostaining indicates an increase in astrocyte population **(J)** and S100β expression is confined to the SVZ and hilum regions **(K)**. The GFAP immunostaining does not coincide with the S100β in the merged images **(D,H,L)**. However, at P2 some progenitors are labeled with both GFAP and S100β (arrows; **P**). DAPI (blue) clearly indicated the brain areas focused **(A,E,I)**.

The article "Differential temporal expression of S100β in developing rat brain" was retracted in 2023. Reasons: unreliable data; unreliable results or conclusions; concerns about the images.

### S100β + GFAP

The dual immunolabeling with S100β and GFAP facilitated to investigate the association of S100β with astrocytes. The results revealed that S100β gets associated with astrocytes only during 2nd postnatal week. While throughout the embryonic life, S100β was expressed only by the progenitor cells and radial glia lining the VZ and SVZ and did not co-expressed GFAP (Figures 5A–H). Although GFAP expression was first seen at E16 (Figure 5F), there was no co-localization with S100β (Figure 5H). Even at birth, the S100β expression was very much specific and confined only to the SVZ and not associated with differentiated astrocytes at all (Figures 5I–L). Subsequently, at P2 and P5 some of the progenitors expressing S100β also expressed GFAP, similar to the observation made through nestin and S100β co-labeling (Figures 5M–P, 6A–D). Even stem astrocytes forming glial tubes, depicting chain migration also co-expressed S100β and GFAP. With further development, by P12 onwards, the S100β expression was downregulated both in the SVZ and SGZ and was recorded in the cell bodies of GFAP labeled astrocytes in the merged images (Figures 6H,L). The results finally indicate that the astrocytes express both S100β and GFAP at maturity with contrasting localization, S100β in the cell soma and the GFAP in the processes of the mature astrocytes (Figures 6E–L).

**Figure 6:** **Dual immunofluorescence staining with GFAP and S100β reveal the association of S100β with mature astrocytes**. DAPI (blue; **A,E,I**), GFAP (green; **B,G,K**) and S100β (red; **C,F,J**). The astrocyte population increases further from P5 to P21 as revealed by GFAP staining **(B,G,K)**. S100β expression was detected in the SVZ at P5 but was found to be associated with the GFAP+ astrocytes at P15 and P30 in hippocampus. The merged images indicate no incidence of co-labeling throughout the period of study **(D,H,L)**. In mature astrocytes the S100β expression was located in the cell soma while GFAP in the processes **(H,L)**.

## Discussion

The epithelial-columnar RG cells form a massive cell system that dominates the early embryonic CNS. They have been accepted for long as mere transitional forms of precursors of astroglia, expressing many glial markers and performing special function of guidance in neuronal migration (Webster and Astrom, 2009). Schematic representation of various cell types generated along the VZ and SVZ in embryonic and postnatal life with a comparison of various developmental milestones in rat and human brain is depicted in Figure 7. The present study supports the stem cell nature of these RG cells expressing nestin, a well established neuronal stem cell marker, throughout the period of CNS development and disappears when they lose their progenitor nature with time. In addition to nestin, both primary progenitor/neuroepithelial stem cells and radial glia/secondary progenitor cells lining the VZ and SVZ were also expressing S100β. Further, both nestin and S100β expression coincided perfectly in the merged images. Thus we propose and demonstrate that S100β can be used as a progenitor marker because of its expression all through the proliferative phase of the progenitors. No other cells at this stage expressed S100β. Once the progenitors loose the capacity to divide and subsequently differentiate into mature cells, S100β is down regulated. We have further noted that the timing of transformation of the radial glia into the mature astrocytes coincides well with the down-regulation of S100β and the disappearance of radial glial fibers. The protein is re-expressed in astrocytes at maturation during 2nd to 3rd postnatal week in rats. It is thus advocated that S100β is a potential progenitor cell marker in the developing nervous system. S100β has been commonly used as a marker of Bergmann glia and white matter astrocytes in the cerebellum of adult mice (Landry et al., 1989). Hachem et al. in 2007 reported its expression in embryonic mouse cerebellum and SVZ and characterized its transient expression in radial glial precursors as a feature of Bergmann cell gliogenesis.

The article "Differential temporal expression of S100β in developing rat brain" was retracted in 2023. Reasons: unreliable data; unreliable results or conclusions; concerns about the images.

**Figure 7:** **Schematic representation of various cell types generated along the VZ and SVZ in embryonic and postnatal life with a comparison of various developmental milestones in rat and human brain**. NEPs = Neuroepithelial cells; RGs = Radial glial cells; SVZ = Subventricular Zone; VZ = Ventricular Zone; wk = Week; BBB = Blood Brain Barrier.

GFAP as RG marker is becoming controversial because of the non-consistent and regionally variable reports in various mammals (Dahl et al., 1981; Schnitzer et al., 1981). For long time the RGs are considered as the precursors of astrocytes and are believed to transform into GFAP expressing astrocytes during early postnatal life in all domains of CNS (Cameron and Rakic, 1991; Marshall et al., 2003; Kriegstein and Alvarez-Buylla, 2009). However, adult NSCs in the SGZ lining the dentate gyrus have long radial processes and express both nestin and GFAP and are called as stem astrocytes, while non-stem astrocytes express only GFAP (Seri et al., 2004; Steiner et al., 2006).

During early postnatal life from P2 to P12, the astrocytes co-expressing nestin and GFAP are seen forming the glial tubes in the neocortical SVZ and also lining the SGZ, indicating the stem cell nature of these so called stem astrocytes. Such Nestin and GFAP co-expressing astrocytes were completely absent throughout the embryonic life and also around birth. Additionally, the cells forming the glial tubes simultaneously expressed S100β and Nestin confirming their proliferative potential. It is thus possible that the RGs that populate the SVZ during late embryonic life till birth are subsequently transformed into stem astrocytes, which then continue to generate neurons. This notion is supported by the investigations made by using nestin-GFP mice and has suggested that the nestin expressing progenitors are converted from astrocytes to neuronal cells (Filippov et al., 2003; Fukuda et al., 2003; Kronenberg et al., 2003). Tramontin et al. (2003) were also of the opinion that the SVZ RGs are abundant around birth and disappear almost completely during first 2 weeks of postnatal life and replaced by adult SVZ astrocytes having proliferative potential which forms glial tubes that are important for chain migration of neuroblasts (Doetsch et al., 1999; Peretto et al., 2005; Bonfanti and Peretto, 2007). Dahl et al. (1985) also reported the association of GFAP with RG during their late stages of differentiation into astrocytes in rodents.

S100β is a highly soluble protein implicated in the initiation and maintenance of a pathological, glial-mediated pro-inflammatory state, and its presence in biological fluids is a well-established biomarker for severity of neurological injury and prognosis for recovery (Ralay Ranaivo et al., 2006). In contrast to the vast literature available indicating S100β expression in majority of glial cells, i.e., astrocytes, ependymal cells, oligodendrocytes, microglia and Schwann cells in various species (Dyck et al., 1993; Rickmann and Wolff, 1995; Adami et al., 2001; Romero-Alemán Mdel et al., 2003; Vives et al., 2003; Deloulme et al., 2004), the present study evidence the specific astrocytic localization on the basis of the observations made with the dual immunolabeling with GFAP, with S100β expressed in the cell body and the GFAP in the processes of the mature astrocytes. Such astrocyte specific localization has also been mentioned in post-mortem human brains from Alzheimer’s and Down’s syndrome patients (Boyer et al., 1991; Wunderlich et al., 1999; Deloulme et al., 2004). Savchenko et al. (2000) also recommended S100β as one of the most specific and reliable markers for astrocytes. However, there are reports mentioning distinct subpopulation of cells with astrocytic morphology in adult brain, immunopositive for either S100β or GFAP (Steiner et al., 2007). Our study reveals no such distinct S100β positive astrocytic population in the post-weaned rat hippocampus, rather astrocytes expressing both S100β and GFAP with contrasting localization, S100β in the cell soma and the GFAP in the processes of the mature astrocytes. Thus the contrasting localization of S100β in GFAP expressing astrocytes can be well correlated with the mature status of the astrocytes, while its co-expression with nestin could be easily interpreted as the stem/proliferative potential of the cells. These results find support from the observations made in the adult mouse brain, where S100β is not expressed in the bipolar GFAP expressing cells present in the Sub granular layer (SGL) and SVZ involved in adult neurogenesis (Filippov et al., 2003; Deloulme et al., 2004; Garcia et al., 2004). Raponi et al. (2007) also documented that S100β is a late marker of astrocyte development and is expressed long after GFAP and characterize a mature stage. Further by using S100β EGFP transgenic mice, they also demonstrated that the onset of S100β expression in astrocytes is associated with the loss of their potential to form neurospheres. Further Raponi et al. (2007) were of the opinion that the S100β expression defines a state in which GFAP expressing cells loose their stem cell potential and acquire a more mature developmental stage, thus the GFAP and Nestin co-expressing progenitors have been shown to be negative for S100β (Filippov et al., 2003). As per Seri et al. (2004) horizontal but not the radial astrocytes could be stained with S100β. Most of these studies, *vide supra*, were carried out in adult system. Our results in the developing system clearly contradicts the above findings on the basis of the clear co-expression of S100β with Nestin in all the nestin+ progenitors throughout the embryonic and early neonatal life, which gradually disappears and reappears in the mature astrocytes. Intracellular S100β acts as a stimulator of cell proliferation and migration and inhibitor of apoptosis and differentiation (Donato et al., 2009). Thus the dynamic expression of S100β in both the NSCs and RGs during embryonic and early neonatal life is associated with its proliferative potential and migration of undifferentiated neuroblasts and astrocytes. Once the NSCs and RGs loose the potential for proliferation, the S100β expression is repressed, thus helping the cells in proliferation.

The article "Differential temporal expression of S100β in developing rat brain" was retracted in 2023. Reasons: unreliable data; unreliable results or conclusions; concerns about the images.

This study thus provides the first clear evidence of S100β expression throughout the period of neurogenesis and early gliogenesis in the developing brain explaining its suitability as a radial progenitor cell marker.

## Conflict of Interest Statement

The authors declare that the research was conducted in the absence of any commercial or financial relationships that could be construed as a potential conflict of interest.
